The article "Link Security Situation Identification Method Based on the Ad Hoc Network of Medical Units" was published in 2022. Journal: Comput Math Methods Med.

# Link Security Situation Identification Method Based on the Ad Hoc Network of Medical Units

**DOI:** 10.1155/2022/3735016

**Published:** 2022-05-06

**Authors:** Yifu Zeng, Qingquan Chen, Ling Yao, Jiajing Zhuang, Zhixuan Huang, Shuhan Huang, Honghua Zeng, Riguang Zhong

**Affiliations:** ^1^The Second Affiliated Hospital of Fujian Medical University, China; ^2^The School of Public Health, Fujian Medical University, China; ^3^The School of Clinical Medicine, Fujian Medical University, China; ^4^Zhongshan College of Dalian Medical University, China; ^5^AngeLong (Fujian) Medical Technology Co., Ltd., China

## Abstract

In order to strengthen the management and security status monitoring of the internal network of medical units and make up for security vulnerabilities in time, an ad hoc network link security situation identification method is proposed. According to the architecture of the ad hoc network, it is analyzed that it has the advantages of strong persistence and its own protocol. Combined with the data of detection equipment and security log, the hierarchical acquisition model is used to obtain the situation elements such as port scanning attack and flood attack. The transmission rate factor, forwarding rate factor, dispersion factor, and node aggregation factor are regarded as eigenvectors. We determine the relationship between identity, difference, and opposition, identify the security situation through the description of the node state, and conduct quantitative processing to obtain the final identification result. The experimental results show that the weight value of this method is the same as the standard weight, which can identify the security situation level, obtain the specific situation value, and present a more intuitive identification result.

## 1. Introduction

In recent years, the informatization of medical institutions has become a general trend. On the one hand, it is the rapid development of Internet medical treatment, and on the other hand, the informatization and standardization of medical procedures are strengthened. Informatization not only effectively improves the work efficiency of medical units and meets the needs of patients for medical treatment but also lays a good foundation for the sustainable development of units. At the same time, information construction and development are also facing many network security problems, including patients' personal privacy information being stolen and external hackers invading the internal network. Traditional medical units have very weak intention of Intranet security construction, and patient information is more likely to be used illegally and cause great losses. Therefore, the network security identification and monitoring of the internal self-organizing network in medical units have become part of the research hotspots.

The article "Link Security Situation Identification Method Based on the Ad Hoc Network of Medical Units" was published in 2022. Journal: Comput Math Methods Med.

A network link security situation awareness method based on the Radial Basis Function (RBF) neural network was proposed [1]. The neural network model is optimized by a hybrid hierarchical genetic method to improve global search ability and realize security situation awareness. A fuzzy reasoning method was proposed [2] to realize automatic identification of security situation and deduces link attack correlation and risk.

The above methods lay a good foundation for the research of network link situation security identification but also have some shortcomings. For example, the data source is single, and there is no quantitative processing of the identification results, so the results obtained are not intuitive. In view of the above defects, this paper uses set pair analysis theory to identify the network link security situation. Set pair analysis is an algorithm dealing with the quantitative similarity and difference of uncertain systems [3], in which set pair represents a set of correspondence between two sets which have some relation. The idea of situation identification by this method is to analyze the system composed of set pair [4], find out the expression of connection number and the calculation method of identity and difference, and analyze the set pair situation, so as to obtain the security situation of the network link [5]. Because this method can deal with the uncertainty caused by fuzzy, random, and incomplete information, it is especially suitable for the security situation identification of the internal network of medical units.

## 2. Analysis on the Structure and Characteristics of the Ad Hoc Network in Medical Units

In traditional data center construction, there are usually three layers of network structure, which are called access layer, aggregation layer, and core layer. As shown in Figure 1, the access layer switches generally connect to servers and aggregation layer switches connect to access layer switches and generally provide other services, such as firewalls, IPS, and WAF. Generally, the aggregation layer is the demarcation point between L2 and L3. The L2 network is below the aggregation switch, and the L3 network is above the aggregation switch. Core layer switches generally provide high-speed forwarding of packets in and out of the data center and simultaneous forwarding of communications between multiple aggregation switches in the data center.

In this system, the physical layer uses the transmission medium to provide the physical connection for the access control and realizes the encoding, decoding, receiving, and sending of signals. The link layer is responsible for establishing and maintaining data connections, as well as wireless links for management and traffic control.

The article "Link Security Situation Identification Method Based on the Ad Hoc Network of Medical Units" was published in 2022. Journal: Comput Math Methods Med.

## 3. Network Link Security Situation Identification Based on Set Pair Analysis

### 3.1. Situation Element Acquisition

Situation elements are obtained from logs and warning events of various anomaly detection devices and security devices, and attack types are divided into network detective, host service, and network resources [6, 7]. Specific attacks are as follows:

1. Port scan

Ports belong to the connection terminal, play the role of a carrier, and also are the main object of attack and scanning. When scanning begins, the attacker transmits a large number of data packets to the host and analyzes the running and open ports on the target host in combination with the receiving and response status. Because all systems have certain security vulnerabilities, attackers can research targeted attack strategies according to the scanning results.

(2) UDP flood

The User Datagram Protocol (UDP) flood attack is also called a flood attack. This attack uses UDP, which eliminates the need for connection construction and authentication during data transmission. During the attack, the attacker sends abnormal data packets in batches, which consumes the network resources of the attacked host by occupying bandwidth. In addition, the host is too busy processing data packets to take care of normal connections, resulting in system crash [8].

(3) Web DoS attack

A Denial of Service (DoS) attack transmits massive data in correct format but not within normal services to the host. The host does not distinguish normal services from abnormal services. Due to limited resources, some normal business was refused [9]. However, due to the gradual improvement of server performance, a small number of packets of attackers can no longer damage the server, so the attackers jointly send DoS attacks to the host, which is the so-called distributed denial service attack.

(4) Illegal access request

Illegal request indicates the network access that does not comply with communication policies and rules. Collecting security data of this part is of great significance for network link security situation identification.

With the increase in the number of users, the network data is gradually huge. How to extract effective information from the huge network system is the basis of situation identification. To this end, the situation element acquisition framework is constructed as follows.

In this paper, the hierarchical situation element acquisition model is used to analyze the situation elements, as shown in Figure 2. The acquisition method is divided into global analysis and local analysis and follows the principle of local before the whole to realize the acquisition of elements.

The article "Link Security Situation Identification Method Based on the Ad Hoc Network of Medical Units" was published in 2022. Journal: Comput Math Methods Med.

### 3.2. Feature Vector Property Selection

The main goal of network link security situational awareness is to obtain characteristic information of network operation [10], analyze the relationship between these information, and obtain the degree of influence on network security situation. In view of the above common attack events, the following factors are selected as feature vector attributes in this paper.

1. Transmittance factor

The transmit rate factor can determine how many packets a node generates and transmits per unit time. Assume *S*_*k*_(*t*) represents the number of data packets generated by node *k* within time slot *t*. When the network environment is relatively stable, *S*_*k*_(*t*) is also relatively stable. If the average value of *S*_*k*_(*t*) is much higher than *S*_*i*_(*t*), it indicates that node *k* has the possibility of launching DoS attacks. Otherwise, node *k* may fail. The expression of the transmittance factor is as follows:

(1) $$\begin{array}{c} S_{Rk}\left(t\right)=\frac{n\times S_{k}\left(t\right)}{\sum_{1}^{n}S_{i}\left(t\right)}, \end{array}$$

where *n* is the number of sending times.

(2) Forwarding factor

The forwarding rate factor can judge the level of packets forwarded by nodes. Assume that *R*_*k*_(*t*) is the number of packets received by node *k* in time slot *t* and *T*_*k*_(*t*) is the number of packets sent by node *k* at the same time. If *T*_*k*_(*t*) is much higher than the average value of *T*_*R*_(*t*), it indicates that node *k* has the possibility of launching black-hole attacks. The calculation formula of the forwarding factor is as follows:

(2) $$\begin{array}{c} S_{Tk}\left(t\right)=\frac{n\times \left(T_{k}\left(t\right)/R_{k}\left(t\right)\right)}{\sum_{n}^{n}T_{R}\left(t\right)/R_{k}\left(t\right)}. \end{array}$$

(3) Data source dispersion factor

Data source dispersion can evaluate data dispersion. Assume that *R*_*Nk*_(*n*) represents the number of neighbor nodes in the first *n* packet received by node *k* and *N* represents the total number of nodes [11]. A large number of *R*_*Nk*_(*n*) indicates that nodes are suspected of launching hexenbiest Sybil attacks. The description formula of the discrete factor is as follows:

(3) $$\begin{array}{c} S_{Dk}\left(n\right)=\frac{R_{Nk}\left(n\right)}{N}. \end{array}$$

(4) Node aggregation factor

The aggregation factor is an indicator to measure the concentration degree of the node's next hop. Assume that *S*_*kj*_(*n*) represents the total number of the first *n* packets transmitted by node *k* to the *j-*th neighbor node and *S*_*pk*_(*n*) represents Max (*S*_*Pk*1_(*n*), *S*_*Pk*2_(*n*), *S*_*Pk*3_(*n*), ⋯). If the value of *T*_*Ak*_(*n*) is lower than the average value of *T*_*NA*_(*n*), the node *k* is suspected of launching attacks, and the definition is as follows:

(4) $$\begin{array}{c} T_{Ak}\left(n\right)=\frac{S_{Pk}\times n}{T_{NA}\left(n\right)}. \end{array}$$

The features of ad hoc network link state data are extracted by the above factors, and the network link security situation identification model is constructed based on these features.

The article "Link Security Situation Identification Method Based on the Ad Hoc Network of Medical Units" was published in 2022. Journal: Comput Math Methods Med.

### 3.3. Security Situation Identification Model

The node records and distinguishes all received and sent data packets in time slot *t*, and the data information vector passing through the node in this period is expressed as *D* = (*d*_1_, *d*_2_, *d*_3_, ⋯*d*_*n*_). The data vector *D* and the elements in the feature information vector set *M* = {*M*_1_, *M*_2_, ⋯, *M*_*i*_} constitute identical-discrepancy-contrary system (IDCS). Suppose that the relation between *D* and *M*_*k*_ in the *x*-th component is expressed as *μ*_*x*_^*k*^; according to the set pair analysis principle, the equation for describing the system is as follows:

(5) $$\begin{array}{c} \mu_{x}^{k}=a_{x}^{k}+b_{x}^{k}i+c_{x}^{k}j. \end{array}$$

In the formula, *a*_*x*_^*k*^  represents the degree of sameness between the data vector *D* and the feature vector *M*_*k*_  in the *x*-th component; the larger the value is, the higher the value is and the more similar the two data are. *b*_*x*_^*k*^ represents the degree of difference between the two components; the larger the value is, the stronger the uncertainty degree is and the larger the value is. *c*_*x*_^*k*^ represents the degree of opposition; a large value indicates a high degree of contrast between information *i* and *k*.

If the *x*-th component is a continuous variable, the set pairs of vector *D* and *M*_*k*_ on the *x*-th component can be expressed as

(6) $$\begin{array}{c} \varphi_{x}=\frac{\left|z_{x}^{d}-z_{x}^{m}\right|}{\left(z_{x}^{d}+z_{x}^{m}\right)}, \end{array}$$

where *z*_*x*_^*d*^  and *z*_*x*_^*m*^ , respectively, represent the value of the *x*-th component vector *D* and *M*_*k*_. Take *ε*_same_ and *ε*_contrary_ as set pair potential critical values, and 0 ≤ *ε*_same_ < *ε*_contrary_ ≤ 1 [12]. The relationship between the degree of identity, difference, and opposition in the expression of the degree of connection is shown in Table 1.

If the *x*-th component vector is a discrete variable, when *z*_*x*_^*d*^ = *z*_*x*_^*m*^, then *a* = 1, *b* = *c* = 0; otherwise, *c* = 1, *a* = *b* = 0, so the sensitivity of *x* to the whole vector is *ω*_*x*_. Combined with the identical-conflicting properties of the set pair analysis, the degree of connectedness can be divided into the sum of a finite number of connectedness factors. The discrete multivariate relation degree of the data vector *D* and the feature information vector *M*_*k*_ is expressed as follows:

(7) $$\begin{array}{c} \mu^{k}=\frac{\omega_{x}\mu_{x}^{k}+\omega_{2}\mu_{x}^{k}+\cdots +\omega_{x}\mu_{x}^{k}+\cdots +\omega_{n}\mu_{n}^{k}}{n}. \end{array}$$

The following formula can be obtained from equation (7):

(8) $$\begin{array}{c} \mu^{k}=\frac{1}{n}\left[\omega_{1},\omega_{2},\cdots ,\omega_{n}\right]\left[\begin{array}{ccc} a_{1} & b_{1} & c_{1}\\ \vdots & \vdots & \vdots \\ a_{n} & b_{n} & c_{n} \end{array}\right]\left[\begin{array}{c} 1\\ i\\ j \end{array}\right]. \end{array}$$

Because there is an inverse relationship between the identical degree and degree of opposition, so *j* < 0, therefore equation (7) can also be converted into the following form:

(9) $$\begin{array}{c} \mu^{k}=\frac{\sum_{x=1}^{n}\omega_{x}\left(a_{x}^{k}-\left|j\right|c_{x}^{k}\right)+\sum_{x=1}^{n}\omega_{x}b_{x}^{k}i}{n}, \end{array}$$

where ∑_*x*=1_^*n*^*ω*_*x*_(*a*_*x*_^*k*^ − |*j*|*c*_*x*_^*k*^)/*n* and ∑_*x*=1_^*n*^*ω*_*x*_*b*_*x*_^*k*^*i*/*n* represent the determined and undetermined parts of the correlation expression, respectively. When the known part of the formula is different, a larger value indicates a higher correlation degree, indicating that the two states are more similar. If the determined part is the same [13], a larger value of the undetermined part indicates a lower correlation degree, indicating that the two states have obvious differences; when the same degree of different operating states is lower than the difference degree, that is, 1/*n*∑_*x*=1_^*n*^*ω*_*x*_(*a*_*x*_^*k*^ − *b*_*x*_^*k*^) < 0, in this case, the node tends to be in an uncertain state. The *ω* value is calculated, and the connection degree of each element in the data vector and feature information vector set is calculated, respectively; *μ*^*x*^ = Max (*μ*^1^, *μ*^2^, ⋯, *μ*^*l*^); then, the network link state tends to be in the *x*-th state in the feature vector set.

The article "Link Security Situation Identification Method Based on the Ad Hoc Network of Medical Units" was published in 2022. Journal: Comput Math Methods Med.

We set the reference feature vector *S* = {*R*_1_, *R*_2_, ⋯, *R*_*i*_}, where *R*_*i*_(*i* = 1, 2, ⋯, *l*) represents the proportion of the total number of nodes in the *i*-th state in the feature vector to the total number of nodes; the situation vector to be measured is *s* = {*r*_1_, *r*_2_, ⋯, *r*_*i*_}, where *r*_*i*_(*i* = 1, 2, ⋯, *l*) describes the proportion of the *i*-th state node in the whole node [14]. The security situation value of the network link to be tested can be expressed by the formula of network security entropy:

(10) $$\begin{array}{c} \rho =\frac{\sum_{i=1}^{l+1}\partial_{i}\times {\left(R_{i}-U_{i}\right)}^{2}}{\sum_{i=1}^{l+1}\partial_{i}\times {\left(R_{i}-r_{i}\right)}^{2}}, \end{array}$$

where *U*_*i*_ represents the percentage of the number of nodes in the *i*-th state in the total number under the condition of absolute insecurity and *∂*_*i*_ represents the weight of components. The higher the *ρ* value is, the more secure the network link is, and the preliminary identification of the network link security situation is realized.

In a statistical period, each attack event may have multiple events *e*. The attack hazards of multiple events of the same type will be accumulated when the security factor situation is calculated. Therefore, the quantitative identification formulas of network detective security element situation *P*_*D*_, host service element situation *P*_*S*_, and resource element situation *P*_*N*_ are as follows:

(11) $$\begin{array}{c} P_{D}=h_{D}\times \underset{e\in E_{t}}{\sum }\left(H_{e}\times I_{e}\right), \end{array}$$

(12) $$\begin{array}{c} P_{S}=h_{S}\times \underset{e\in E_{t}}{\sum }\left(H_{e}\times I_{e}\right), \end{array}$$

(13) $$\begin{array}{c} P_{N}=h_{N}\times \underset{e\in E_{t}}{\sum }\left(H_{e}\times I_{e}\right), \end{array}$$

where *h*_*D*_ represents the situation factor of network detective security factor, *h*_*s*_ represents the situation factor of host service factor, *h*_*N*_ represents the situation factor of resource factor, *H*_*e*_ represents the possibility of attack, *I*_*e*_ represents the attack intensity, and *h*_*t*_ represents the attack harm factor.

## 4. Simulation Experiment and Result Analysis

In order to prove the performance of the proposed network link security situation recognition method, a network as shown in Figure 3 is constructed for the simulation experiment. This includes network facilities such as server nodes, routers, firewalls, and switches. The node performance information can be collected in real time to obtain the performance information of each link.

The server weight data and link weight values in Figure 3 are shown in Tables 2 and 3, respectively.

As can be seen from Tables 2 and 3, the weight values of server topology and main link topology are the same as the corresponding standard weights, respectively, indicating that network link security situation has good identification performance.

In order to facilitate the administrator to make decisions, the identification results are quantified. In the situation calculation of security elements, hazard coefficients of various attack events are determined based on management experience, as shown in Table 4.

The article "Link Security Situation Identification Method Based on the Ad Hoc Network of Medical Units" was published in 2022. Journal: Comput Math Methods Med.

The recognition results of the proposed method are compared with the expected results, as shown in Table 5.

As can be seen from Table 5, there is no significant difference between the security situation value identified by the proposed method and the expected output value. Only in the ninth simulation process, there is a certain deviation in the classification of security level, which is due to the existence of certain interference information in the process of situation factor acquisition.

## 5. Discussion

In recent years, with the rapid development of Internet, medical care and health service informatization level gradually strengthens while the risk of network security increases as well. The medical unit network is vulnerable to all kinds of network attacks, which not only gives rise to the information leakage of patient privacy but also hinders the further development of medical informatization. It has become a hot research topic currently.

In this paper, a link security situation identification method is proposed by analyzing the internal network structure of medical units and combining with set pair analysis theory. The simulation results show that the proposed model can well identify the risk levels of different links in the internal network of medical units and provide valuable suggestions for preventing network attacks.

Note that if predictive control algorithms in this field [15–17] may be implemented, the network security and managers' decision-making ability would be further enhanced.

## 6. Conclusion

In order to strengthen network security and improve managers' decision-making ability, a research on security situation identification based on set pair analysis is proposed. By collecting situation elements and extracting features, a situation recognition model is established. Simulation results show that there is little difference between the security situation values identified by this method and the expected output values. However, the acquisition process is completed manually. In the future research, automatic acquisition and preprocessing of situation elements will be realized to further reduce the identification of interference factors. In addition, the experimental environment is limited, so whether the situation recognition method based on set pair analysis can be applied to the internal network of large-scale medical units remains to be further studied.

## Figures and Tables

**Figure 1:** Self-built network structure diagram of medical units.

**Figure 2:** Framework diagram of hierarchical situation identification elements.

**Figure 3:** Topology diagram of simulation experiment.

The article "Link Security Situation Identification Method Based on the Ad Hoc Network of Medical Units" was published in 2022. Journal: Comput Math Methods Med.

**Table 1:** Coefficient and set pair relations.

Set pair potential distribution	Value of *a*, *b*, and *c*
0 ≤ *φ*_*n*_ ≤ *ε*_same_	*a* = 1, *b* = *c* = 0
*ε*_same_ ≤ *φ*_*n*_ ≤ *ε*_contrary_	*b* = 1, *a* = *c* = 0
*ε*_contrary_ ≤ *φ*_*n*_ ≤ 1	*c* = 1, *a* = *b* = 0

**Table 2:** Server topology weight data.

Server type	Topology weight	Standard weight
Server 1	0.3	0.3
Server 2	0.3	0.3
Server 3	0.4	0.4

**Table 3:** Main link topology weight.

Link	Topology weight	Standard weight
Link 1	0.4	0.4
Link 2	0.2	0.2
Link 3	0.4	0.4

**Table 4:** Attack event harm coefficient.

Attack event	Attack type	Harm coefficient	Note
Port scan	Internet detective	2	Attacks do less damage in the early stages
UDP flood		3	A large number of data packets impact host services
Web DoS	Host service	4	Resources are valuable and the attack is harmful
Illegal request		2	Blocking events that control access to the system
Broadcast	Network resource	2	A network storm occurs, occupying bandwidth

**Table 5:** Comparison of experimental results.

Experiment number	Actual threat level	Expected threat level	Actual output value	Expected output value
1	High	High	0.78	0.77
2	High	High	0.75	0.86
3	High	High	0.70	0.71
4	Medium	Medium	0.68	0.68
5	Medium	Medium	0.62	0.62
6	Medium	Medium	0.57	0.56
7	Medium	Medium	0.51	0.51
8	Low	Low	0.45	0.45
9	Medium	Low	0.52	0.52
10	Low	Low	0.38	0.38

## Data Availability

Data can be available on request from the authors due to privacy/ethical restrictions.
